# Obstetrics Nursing and Medical Health System Based on Blockchain Technology

**DOI:** 10.1155/2021/6631457

**Published:** 2021-03-05

**Authors:** Baolin Sun, Zhihui Lv, Qin Li

**Affiliations:** Department of Obstetrics, Affiliated Hospital of Qinghai University, Xining 810000, Qinghai, China

## Abstract

Blockchain, as an emerging force transforming the Internet, has applications in finance, logistics, public services, and other fields. It will also have a huge impact on the medical and health industry. The salient features of blockchain technology include guaranteeing information security and user privacy, decentralization, without the involvement of third-party trust institutions, and being able to establish a high-value input and output two-way system, which has a very important application space in obstetric care, medical, and health. The traditional medical and health system is far from being able to meet the information exchange between doctors and individuals. Therefore, building an interconnected obstetric care and health system based on blockchain technology is the direction of future obstetric care and medical development. This paper has conducted an in-depth study of the obstetric care medical health system, with the help of the Internet of Things, blockchain, and other technical means; the purpose is to realize the sharing and security of medical data and to break the limitations of traditional user information. This paper builds a medical electronic health record system model and a hybrid consensus model based on blockchain technology to realize the safety and transparency of patients' personal medical information data and achieve two-way communication and interconnection of information between doctors and patients. This paper analyzes the current status of domestic and foreign medical and health systems and the blockchain-based medical electronic health record system. It is concluded that the domestic investment in medical and health in 2018 was as high as 113.2 billion yuan, and the entire investment scale is continuously expanding. Pay attention to the health system. In the future, the obstetric care and medical health system based on blockchain technology will surely be realized and improved.

## 1. Introduction

With the development of cities and the improvement of people's living standards, more and more people have begun to pay attention to their personal health, especially paying more attention to maternal health care. My country's medical and health demand continues to grow. With the promotion of Internet technology, “Internet of Things + Medical” has become an inevitable trend in the pharmaceutical industry. In addition, the establishment of a medical and health system based on the blockchain is also a general trend.

As a kind of information technology, blockchain can be used as a shared ledger distributed in scattered points, using a consensus mechanism to perform encryption algorithm calculation results and finally achieve point-to-point information transmission. Its most prominent feature is as follows: in the data link, it can track the data source and cannot modify any data at will, with high transparency and openness. In summary, it achieves data security and transparency and provides trust guarantee for the use of blockchain. The combined use of blockchain and obstetric care and medical care is well suited to the characteristics of decentralization and promotes trust and cooperation between multiple subjects.

Huang H designed a health care system (HES) framework that collects medical data from WBAN, transmits the medical data through a wide range of wireless sensor network infrastructure, and finally publishes it to the wireless personal area network through the gateway. In addition, HES involves a group of transceiver model solutions to achieve key distribution and secure data transmission, matrix-based homomorphic encryption to ensure privacy, and an expert system that can analyze scrambled medical data and automatically feed back the results. Theoretical and experimental evaluations were conducted to prove the safety, privacy, and improved performance of HES compared to current systems or solutions. However, the further prosperity of electronic/mobile healthcare still faces many challenges, including information security and privacy protection [1]. In order to promote learning in health system science and add value to the health system, Gonzalo et al. tried to determine the true roles of students in a series of clinical settings and explored the value of the students who fulfilled these roles. From 2013 to 2015, they conducted a series of on-site visits and leadership interviews at clinical sites (*n* = 30). Thematic analysis is used to determine the tasks and benefits of incorporating students into the interprofessional nursing team. Types of system roles include direct patient benefit activities, including monitoring patient progress and facilitating access to resources through the care plan, and clinical benefit activities, including promoting coordination and improving clinical processes. The perceived benefits include enhancing the value of the clinical mission and enhancing student education. These results clarify a framework for student roles that can enhance learning and add value to the health system. However, the educational plan that seeks to include students in the role of the system has not been well described [2]. Lemieux aims to explore the value of blockchain technology as a solution for creating and maintaining trustworthy digital records and proposes the limitations, risks, and opportunities of this approach. Methodological approaches involve the use of requirements embedded in records management and digital preservation standards, in particular ISO 15489, ARMA's recognized record-keeping principles, ISO 14721, and ISO 16363, as a common assessment framework based on risk assessments for developing countries' land registration systems of the specific proposed implementation of blockchain technology. The analysis results show that assuming appropriate security architecture and infrastructure management control measures, blockchain technology can be used to solve current and short-term issues related to information integrity. However, it cannot guarantee the reliability of the information from the beginning, and it will be subject to some limitations as a long-term solution to provide reliable information [3].

The innovations of this paper are as follows: (1) This paper uses a combination of quantitative and qualitative methods, which is well reflected in the third part of the mixed consensus mechanism model. (2) This paper uses a combination of theoretical analysis and countermeasure research. While establishing model analysis and giving countermeasures and suggestions, this method runs through this paper. (3) This paper uses the hash algorithm and Merkle tree, data sharing, and lattice algorithm, which is for medical electronics based on blockchain. The health record system EHRS has been fully analyzed.

## 2. Method of Obstetric Care and Medical Health System Based on Blockchain Technology

### 2.1. Overview of Blockchain Technology

The concept of blockchain was proposed by Nakamoto in 2008. It was initially mainly used in economic fields such as finance and insurance and then developed into logistics, Internet of Things, public services, and other fields [4]. Its core technology is the consensus mechanism and the application of smart contracts. By using smart contracts, both parties do not need to use a third party for trust guarantee, which solves the problem of trust transactions. Generally speaking, the blockchain system consists of six layers: data layer, network layer, consensus layer, incentive layer, contract layer, and application layer, which can be programmed at various levels [5].

There are three types of blockchains, namely, public blockchains, joint (industry) blockchains, and private blockchains. The scope and objects of application of the three are different [6]. First of all, the public blockchain has the widest scope of application, the least restrictive conditions, and the lowest requirements, and it can adapt to the most extensive blockchain needs. With the characteristics of decentralization, its transaction speed is also the slowest. Secondly, the joint blockchain mainly refers to the blockchain in a certain industry, which has the characteristics of multicentralization, and its data can realize multiparty intercommunication. The most typical one is the hyperledger. The third is a private blockchain. The typical representative is Ant Financial. Its transaction speed is very fast, which can fully guarantee the company's internal information and provide protection for the company's privacy [7, 8]. The feature comparison between the three is shown in Table 1.

The main characteristics of the blockchain are as follows: (1) Decentralization: the application of blockchain does not have unified central management, and its distributed storage can resist hacker intrusion and protect the privacy of data. And there is no need for unified software and hardware facilities, and the requirements for equipment are average. (2) Cannot be tampered with: it is difficult to modify and delete data because of the constraints of the consensus mechanism in the blockchain [9, 10]. (3) Independence: each smart contract is signed independently by both parties to the transaction, without the blessing and guarantee of a third party. It can calculate the contract according to mathematical algorithms such as hash algorithm and automatically complete the transaction and transaction data.

In summary, it has the characteristics of decentralization, nontampering, whole process mark, traceability, collective maintenance, openness, and transparency. If these characteristics of the blockchain can be used well, the problem of decentralized management of medical equipment can be greatly solved. At the upstream end, enterprises and hospitals upload relevant information through an encrypted system, including medical equipment production information, production quantity, and logistics information; at the downstream end, hospitals, and manufacturers use blockchain technology to strengthen communication and strictly control the compliance of medical equipment, required standards, and so on and increase the recognizability of products, which will help hospitals strengthen the daily management, calculation, and inventory of medical equipment.

### 2.2. Hash Algorithm and Merkle Tree

The hash algorithm is a kind of mathematical algorithm, but in fact, it is more like a thought algorithm. It does not have a fixed formula for calculation. It only needs to input information to compress messages of any length into fixed-length information. For any field, it can improve the utilization of storage space, so it is widely used [11]. In addition, another characteristic of the hash algorithm is irreversibility; that is, it is difficult to find the reverse law, which is a very important application for the medical and health field [12].

The Merkle trusted tree is generated to verify the security of information. It is only based on the security of the hash algorithm and can be verified without too many other assumptions. It uses a traversal algorithm to reduce the calculation idea of redundant hash function values and finally obtains a root hash value through layer-by-layer processing of small data blocks. It has a wide range of applications, mainly in information security, so it is very useful to verify the validity of data in the blockchain [13].

### 2.3. Data Sharing and Lattice Algorithm

Obstetric nursing users store all their personal medical information in a distributed database, use the reencryption key in cryptography to encrypt the information [14], and use it for data upload, browsing, and viewing. In a decentralized blockchain technology, there is no need for a third party to act as an agent for data access application and control. To complete the reencryption operation, you only need to add and modify any node in AFS and MIFS [15].

For example, when a doctor needs to view the patient's past medical information, the patient will perform normal encryption processing on the part that the doctor needs to view and at the same time generate a corresponding proxy reencryption key. Then, the patient selects one of the nodes in the list of competing agents and sends the reencryption key to this node, and then the agent reencryption node will complete the reencryption operation and store the ciphertext in the distributed database. Finally, the doctor uses the private key to open the database and consult the relevant information.

The method of using proxy reencryption can effectively realize data sharing and protect users' privacy rights. This process is called the entrustment of rights [16]. The agreement is formulated in accordance with the results of the lattice algorithm.

(1) Generate a random matrix *A* ∈ *Z*_*q*_^*n*^*∗*^*n*^ and select a safe integer *q*, *n*.
(2) Generate a public-private key pair: the public key *pk*=*P*, *P*=*R* − *A*, and *S* ∈ *Z*_*q*_^*n*^*∗*^1^, where *R* and *S* are Gaussian parameters, and then the private key *sk*=*S*.
(3) Encryption algorithm:
  (1) $$\begin{array}{c} c=\left(c_{1},c_{2}\right)=\left(e_{1}A+e_{2},e_{1}P+e_{3}+m\cdot \left[\frac{q}{2}\right]\right). \end{array}$$
In formula (1), *e*_1_, *e*_2_, *e*_3_ are the error parameters.
(4) Decryption algorithm:
  (2) $$\begin{array}{c} m=c_{1}S+c_{2}. \end{array}$$
Determine whether it is 0 or 1 based on the distance from 0.
(5) Reencryption key generation algorithm:
  (3) $$\begin{array}{c} rk_{a⟶b}=\left(P_{B},Q\right),\\ Q=\left[\begin{array}{cc} X & -XS_{B}+E+S_{A}\\ 0 & I \end{array}\right]. \end{array}$$
Among them, *X* is a random matrix and *E* is noise.
(6) Reencryption algorithm:
  (4) $$\begin{array}{c} \left(c_{1}^{\prime },c_{2}^{\prime }\right)=h_{1}\left(A,P_{B}\right)+\left(h_{2},h_{3}\right)+\left(c_{1},c_{2}\right)\cdot Q. \end{array}$$
Among them, *h*_1_, *h*_2_, *h*_3_ are selected from the error distribution.

## 3. Blockchain-Based Obstetric Care Medical Health System Architecture Model

This section is based on the basic architecture and functional modules of the obstetric care medical and health system based on the blockchain. It describes in detail how blockchain technology improves the privacy, security, and integrity of the medical and health system, so as to realize the blockchain and obstetrics' effective integration of nursing care and health systems.

### 3.1. Medical and Health Electronic File System Model Based on Blockchain

#### 3.1.1. Basic Logical Structure

The architecture model of obstetric care and medical health system based on blockchain is designed into three levels: data storage layer, data connection layer, and data application layer [17]. Take the personal electronic medical health file as a blockchain, and all relevant data and information are stored in the distributed ledger of the blockchain. The data is input, updated, and output through the data connection layer to realize data viewing and review. Finally, the intelligent contract is used for data application, and the implementation of the trigger contract completes the operation of the data [18, 19].  Figure 1 shows the characteristics of the blockchain decentralized healthcare system.

#### 3.1.2. Data Storage Layer

The construction of the obstetric care medical health system model based on blockchain technology is based on the way of blockchain for data storage. In a large database, each person's medical and health records are organized into a separate chain. This data link can be updated and added in real time but cannot be modified or deleted. This effectively guarantees the time cohesion, authenticity, and integrity of its health files [20]. Electronic health records are a lifetime of data generated by the physical health of different ages; it mainly records information related to physical examination items and health activities. The time is not fixed. Therefore, the information is not stored at intervals but is updated in real time [21].

For example, when a mother needs obstetric care, which includes prenatal care and postpartum care, every physical examination data will be directly recorded in the mother's personal exclusive blockchain. A complete blockchain is composed of two parts, namely, the initial source module and the additional module. When creating a personal electronic health file for the first time, you need to record the basic information of the individual. After that, each additional physical examination will automatically generate a block and automatically record it in the blockchain.

The blockchain deployment of the data storage layer adopts the private chain method and the public chain method in each case. If a private chain is used, the amount of data is too large, but the number of nodes can be effectively controlled, it can be installed in major database centers, and the feasibility of implementation is enhanced. If the latter method is used, huge computing resources are required. No matter which method is used, a common technical feature of the blockchain is the consensus mechanism, which can ensure the safety and effectiveness of the entire operation process and limit the control and sharing of its data [22].

#### 3.1.3. Data Connection Layer

In the Bitcoin market, blockchain technology is used to test the authenticity, security, and validity of the transaction process [23]. Then in the model of this paper, the application of blockchain can be used to verify the authenticity of the information of both parties in the transaction and the validity of data operations during the transaction. The function of the data connection layer is to integrate all the user's distributed information into a blockchain and select the appropriate node for storage, participate in the real-time update process of data, and ensure that users can effectively access the blockchain [24]. The blockchain nature of the data that cannot be tampered with at will can ensure the integrity and authenticity of the entire data chain and can also see the traceability of all data, giving users certain rights and operability to ensure the authenticity and validity of the data.

In general, all information operations at this level are safe and reliable. Specifically, the starting block of the blockchain in the data connection layer mainly includes the following aspects: first, determine candidate nodes. The user needs to select the applicable candidate node organization information; generally speaking, he will choose the health information data center [25]; second, determine the user role. Users who apply for the first time can choose among three user roles, namely, owner, operator, and manager [26]. Ordinary users generally choose to be the owner and have full operation authority for their own information and data without any restrictions, but they still cannot modify or delete data information. This is also true for the other two roles. The operator role is generally selected as the health manager of the hospital. After having this role permission, you can apply to view and share the relevant information of the patient and increase the relevant case information, provided that the owner is authorized to succeed. Each node in the initial module is a manager, in addition to operating functions, you can also change user roles [27]. To modify the user role, the following conditions should be met: the operator's role modification requires the identification of the operator, and the operator here must belong to a staff member registered by a health service department with a relevant certificate of practice.

The storage process of the blockchain and the transaction storage process of Bitcoin are essentially the same. Both can record detailed operation records and update real-time status. Therefore, it is possible to increase the information storage in the blockchain at a fixed time interval.

Smart contract is one of the important components of the data connection layer. Intelligent contract is a scripting language based on blockchain, which can be triggered by the state change of blockchain, thus realizing the data operation on blockchain. It is an operating system based on the blockchain to verify the identity and trust of both parties in the transaction. It connects the data storage layer and the data application layer in the entire model, is the bridge of the entire process, and is at the core. Smart contracts are also divided into two categories: one is the smart contract that comes with the system and the other is the smart contract form that can be customized to fully meet the transaction needs and personalized characteristics of the transaction subject.

#### 3.1.4. Data Application Layer

The data application layer refers to the data operation of health files according to specific application requirements, such as user authority management and doctor's viewing information authority [28]. In user authority management, the account owner needs to respond to the current authority application of the relevant person and set the content of the personal information file disclosure authority. The specific process is as follows. First, when the operator requests to access the patient's electronic file information, the smart contract will be triggered; the smart contract is mainly used to verify the applicant's identity information by verifying the applicant's digital signature. After the verification is passed, the operator can check whether the permission of the information he needs is open. If it is open, the data operation is successful. If it is not open, it needs to send an application to the owner again and wait for its reply. If you agree, the next step will be taken. Abandon the operation. The user owner can also set the disclosure of some project permissions, such that nonprivate projects can be opened, but for information-sensitive projects, multiple encryption operations are required.

The two core functions of the data application layer are as follows: the first is permission management; the second is data manipulation. In order to realize the convenience of querying electronic medical health files, you can consider developing related applications, such as permission application API or data manipulation API.

### 3.2. Hybrid Consensus Mechanism Model Based on Blockchain

The hybrid consensus mechanism model *HL*1*HL*2 will be represented by a set *N*_1_^*∗*^ and a set *N*_2_^*∗*^, respectively. There are

(5) $$\begin{array}{c} N_{1}^{*}\geq 3f+1. \end{array}$$

Among them, *f* is the maximum number of error nodes within the acceptable range of *HL*1. For the sake of simple calculation, set as

(6) $$\begin{array}{c} N_{1}^{*}=3f+1. \end{array}$$

*HL*2 is the set of complements *HL*1. In the specific operation, move *HL*1 the limited number of authorized representatives at the bottom to the *HL*2 bottom, and select *HL*2 the limited number of authorized representatives at the top to be moved to the middle *HL*1. The formula can be expressed as

(7) $$\begin{array}{c} N_{2}^{*}=\left\lfloor 2f\right\rfloor ,n=\left|\frac{1}{2}f\right|. \end{array}$$

First of all, it is necessary to reorganize the positional relationship between *HL*1*HL*2 the information of, including the server information in the sum, so that they can match each other. Then, sort these servers by number 1−c. Then, according to the requirements of block height and server number, select the current node *R*, which needs to meet the following formula:

(8) $$\begin{array}{c} R=\left(H+c\right)\mathrm{mod}N_{1}^{*}, \end{array}$$

where *H* is the height of the current block.

Again, the remaining nodes *HL*1 in the setting are all 0, and the number is expressed as {0,1,…, *N*_1_^*∗*^ − 1}; as long as there is “upgrade and downgrade,” the random number can be renumbered; the check node *HL*2 in the command is *C*.

The formula of this model needs to be divided into two steps: initiating consensus and confirming consensus. As long as there is a request from a user or hospital operator, *HL*1 will automatically initiate a consensus on the duty node. In the model in this paper, we set Φ the time interval required for a consensus. Then, the value node will upload the received data information together with the digital signature, then form a block after encryption processing, and finally store it in the blockchain.

In the blockchain, the trigger standard of the consensus mechanism is very high. For example, the original block must maintain a high degree of consistency in order to initiate a consensus. And in the process of confirming the consensus, the medical data, server information, *H*, and hash index of all nodes must be consistent, which is quite high for hospitals.

## 4. Obstetric Care and Medical Health System Based on Blockchain Technology

### 4.1. The Current Situation of Domestic and Foreign Medical and Health Systems

#### 4.1.1. Scale of Domestic Medical and Health Industry

Compared with foreign countries, my country's time to attach importance to the medical and health system is much later. However, following the national strategy and the support of national policies, the development of the domestic obstetric care and medical health system is steadily improving. From the data in Table 2, it can be seen that the scale of my country's medical and health industry in 2011 was only 1.7 trillion yuan, and the scale of development was not large enough; however, as can be seen from the line chart in Figure 2, the annual growth rate is very fast, and the growth rate exceeds 10%, even as high as 35% growth rate in 2013. As of the end of 2018, the market size of the domestic medical and health industry was 5.9 trillion yuan, and its scale has expanded several times. It can be seen that my country's medical and health industry has a bright future.

#### 4.1.2. The Scale of Domestic Medical and Health Investment

It can be seen from Table 3 and Figure 3 that my country's domestic healthcare investment and financing scale has shown an upward trend from 2010 to 2018. In 2015, the investment amount was 623 trillion yuan, with an increase of 48%; after 2015, my country's investment in the medical and health field has increased rapidly, and the total investment has expanded several times, which can well represent the domestic medical and health field in my country.

#### 4.1.3. Global Healthcare Investment and Financing

As shown in Table 4 and Figure 4, the financing scale of the global healthcare industry has made a huge leap in 2015 and 2017, and at the same time, financing events have also increased significantly. In 2018, the amount of financing was 158 billion yuan, with a year-on-year increase of 37%. The financing event was 1030, and the increase in financing events was not fluctuating. This shows that the amount of financing in the early years is directly proportional to the occurrence of financing events, while the performance in recent years has shown an irregular state. In the case of a small increase in the number of financing events, the amount of global medical and health financing is still increasing significantly, indicating that for most people the enthusiasm for financing has not diminished and may hold a wait-and-see attitude or increase investment in the same project.

#### 4.1.4. Global and Domestic Financing Changes in the Medical and Health Industry Segments

It can be clearly seen from Table 5 that, in 2018, the investment and financing fields of the global healthcare industry were mainly concentrated in biotechnology, medicine, medical informatization, and medical equipment, with financing amounts of 511 trillion yuan, 278 trillion yuan, and 299 trillion yuan, respectively. The total investment is 295 trillion yuan, and the total number of investment events exceeds 1,000, accounting for 73% of the total.

It can be seen from Figure 5 that the amount of investment in biotechnology far exceeds investment in other fields, and the latter are mainly innovative fields driven by consumer demand. More exploration has not been carried out, such as rehabilitation nursing, bioengineering, and medical tools. The financing situation in these areas is not optimistic.

As can be seen from Table 6 and Figure 6, the domestic investment enthusiasm is still slightly different from the international investment field. The top ones with the highest enthusiasm for domestic healthcare investment are biotechnology, medicine, medical informatization, and primary care. The financing amount is much lower than the global financing amount, which is 119 trillion yuan, 69 trillion yuan, 73 trillion yuan, and 60.9 billion yuan, respectively. Secondly, there is a general investment preference in several areas such as drug sales, medical equipment, medical technology, and consumer medicine.

In general, in the direction of domestic and global medical and health investment and financing subdivisions, science and technology are the main orientation, and technological innovation has shown great advantages in the fields of biotechnology, medical informatization, medicine, and so on. The amount of investment and financing is much higher than that in other fields; in addition, the enthusiasm for investment in consumption or service-oriented fields is not high.

### 4.2. Ehrs Analysis of Medical Electronic Health Record System Based on Blockchain

The purpose of constructing a blockchain-based obstetric care medical health system is to use the advantages of blockchain to solve the shortcomings of the traditional medical system, especially the reading of personal health information data and the security of information data. Traditional medical and health systems have disadvantages such as difficulty in storing information and cumbersome procedures for reviewing information and data verification, and the entire process is prone to data modification and data insecurity. These are not conducive to building a more complete and safe smart medical care.

It can be seen from Figure 7 that, since 2011, my country's nursing hospitals have begun to use standardized EHR on a large scale. By the end of 2017, almost 100% coverage has been completed. This shows the development of the medical data information era and the relatively mature medical data informatization; these can partially solve the storage and access application problems of medical information.

From Table 7 and Figure 8, we can see that different types of hospitals use the basic version of EHR to different degrees, but there is a certain degree of growth every year. The growth rates of small hospitals and rural hospitals are almost the same. Large hospitals and emergency hospitals have increased significantly from 2014 to 2018. The data of the two hospitals in 2018 were 83 and 80, respectively, compared with 28 and 20 in 2014, an increase of more than 60%. This shows that more and more hospitals are also aware of the importance of medical and health data sharing, which brings great convenience to both doctors and patients.

In general, the current application and research of blockchain in the medical field have attracted much attention. The development of blockchain technology has changed the traditional way of centralized storage of medical data, eliminating the auditing role of intermediaries and blockchain technology. It can help doctors, patients, and researchers to authenticate permissions quickly and safely and realize free data access and sharing.

## 5. Conclusions

The paper is mainly to study the construction of obstetric nursing medical health system based on blockchain technology. Through in-depth research on blockchain, it can be effectively applied to the medical health system of obstetric nursing. This paper uses a combination of qualitative and quantitative research methods, an in-depth understanding of the blockchain, combined with the characteristics of the blockchain's decentralization, trustlessness, information security and transparency, and its role in obstetric care and health care. It helps to build a complete medical and health system based on blockchain. The combination of blockchain technology and medical health system forms a new model for the development of information data in the field of the medical word.

In this paper, the hash algorithm and Merkle tree, data sharing, and lattice algorithm are used to construct a blockchain-based medical and health electronic file system model and a blockchain-based hybrid consensus mechanism model and analyze domestic and foreign medical. The current health system and the EHRS analysis of the blockchain-based medical electronic health record system show that there are still information asymmetry and information security issues in the domestic medical health system. The obstetric care medical health system based on blockchain technology can solve these problems well.

In the future, the establishment of this system will strengthen the relationship between doctors and patients and achieve multidirectional communication and information exchange. In the process of in-depth research on the combination of blockchain and the medical field, we also realized that there are still some difficulties in the research topic of this paper. The first is the contradiction between decentralization and centralized management. Although decentralization has advantages, it also has disadvantages, such as the lack of a unified management core, and the system cannot be automatically adjusted or repaired. The second is that the standards of blockchain technology have yet to be improved. The complexity of the blockchain itself, coupled with numerous problems in the medical and health field, has a serious impact on it and restrict the development of the blockchain medical and health system.

## Figures and Tables

**Figure 1:** Blockchain decentralized healthcare system.

**Figure 2:** Scale and growth rate of domestic healthcare industry from 2011 to 2018.

**Figure 3:** China's healthcare financing.

**Figure 4:** Global healthcare financing.

**Figure 5:** Changes in financing of the global health care industry in 2018.

**Figure 6:** 2018 China's medical and health industry sector financing situation.

**Figure 7:** The proportion of basic EHR and standard EHR adopted by nursing hospitals from 2010 to 2017.

**Figure 8:** The percentage of different types of hospitals using basic EHR.

**Table 1:** Comparison of characteristics of public chain, alliance chain, and private chain.

Blockchain characteristics	Public chain	Alliance chain	Private chain
Target the crowd	Anyone	Specific organization	Individual person or entity
Degree of centralization	Decentralization	Polycentric	Centralization
Incentives	Need	Optional	Not needed
Node write	Free to join	Authorization required	Internal control
Transaction speed	3–20 pens/sec	1000–10000 pens/sec	1000–10000 pens/sec
The Internet	P2P network	High-speed Internet	High-speed Internet
Node storage	Personal computer	Specific server	Specific server
Access threshold	Low	Higher	Very high
Application representative	Bitcoin blockchain; Ethereum smart contract	Hyperledger	Ant Financial
Practical field	Digital currency transactions, financial asset transactions, proof of existence, and so on	Transaction within the organization, bank or country clearing, and settlement	Companies, governments, hospitals, and other entities, used as internal information systems

**Table 2:** Scale and growth rate of domestic healthcare industry from 2011 to 2018.

	Industrial scale (trillion yuan)	Growth rate (%)
2011 year	1.7	
2012 year	2	25
2013 year	2.8	35
2014 year	3.5	26
2015 year	3.9	15
2016 year	4.7	18
2017 year	5.2	11
2018 year	5.9	17

**Table 3:** China's healthcare financing.

	Financing amount (100 million yuan)
2010	65
2011	63
2012	75
2013	120
2014	348
2015	623
2016	852
2017	967
2018	1132

**Table 4:** Global healthcare financing.

	Financing amount (100 million yuan)	Event (a)
2011	52	235
2012	73	220
2013	122	336
2014	179	489
2015	392	856
2016	587	1324
2017	985	1291
2018	1580	1030

**Table 5:** Changes in financing of the global healthcare industry in 2018.

	Financing amount (100 million yuan), Number of events	Event (a)
Biotechnology	511	224
Medicine	278	82
Medical information	299	365
Medical equipment	295	372
Technology medical	119	301
Primary care	119	60
Drug sales	28	29
Great health	21	89
Medical finance	29	18
Consumer medical	26	19
Rehabilitation nursing	16	18
Seek medical advice	12	12
Medical tools	6	1
Motherhood	5	17
Medical support	5	12
Seek a doctor	5	8
Biological engineering	2	2
Circulation channel	0.8	1

**Table 6:** 2018 China's medical and health industry sector financing situation.

	Financing amount (100 million yuan), number of events	Event (a)
Biotechnology	119	84
Medicine	69	38
Medical information	73	68
Medical equipment	25.8	76
Technology medical	21.3	37
Primary care	60.9	33
Drug sales	47.3	19
Great health	18.8	44
Medical finance	12.3	6
Consumer medical	24.3	25
Rehabilitation nursing	4.5	11
Seek medical advice	3.8	7
Medical tools	5.2	6
Motherhood	3.3	15
Medical support	2.3	8
Circulation channel	0.6	1

**Table 7:** The percentage of different types of hospitals using basic EHR.

	All hospitals	Small hospital	Rural hospital	Critical access hospital
2014	28	21	21	20
2015	42	39	37	36
2016	59	51	51	52
2017	78	70	70	68
2018	83	81	80	80

## Data Availability

No data were used to support this study.
